The article "The Neutrophil-Lymphocyte Ratio Is Positively Correlated with Aggression in Schizophrenia" was published in 2022. Journal: Biomed Res Int.

# The Neutrophil-Lymphocyte Ratio Is Positively Correlated with Aggression in Schizophrenia

**DOI:** 10.1155/2022/4040974

**Published:** 2022-04-23

**Authors:** Zhu Tong, Jing Zhu, Jia-jia Wang, Yu-jing Yang, Wei Hu

**Affiliations:** Department of Psychiatry, The Affiliated Xuzhou Eastern Hospital of Xuzhou Medical University, Xuzhou, Jiangsu, China

## Abstract

To find biomarkers to assess the risk of aggression, we looked at the association between aggression and levels of body inflammation in patients with schizophrenia. The Modified Overt Aggression Scale (MOAS) score was used to divide the aggressive (*n* = 72) and nonaggressive (*n* = 141) groups. The Brief Psychiatric Rating Scale (BPRS) is a tool for determining the severity of a patient's condition. After measuring the number of inflammatory cells in the peripheral blood, the platelet-lymphocyte ratio (PLR), neutrophil-lymphocyte ratio (NLR), and monocyte-lymphocyte ratio (MLR) were estimated. We investigated the relationship between aggressive behavior, bodily inflammation, and BPRS. Before therapy, the aggressive group's BPRS score, white blood cell (WBC) count, neutrophil count, monocyte count, NLR, and MLR were considerably more significant than the nonaggressive group's. After therapy, statistically significant variations in total BPRS score and neutrophil count between the two groups. According to correlation analysis before and after treatment, aggressive behavior was positively connected with neutrophil count, NLR, and BPRS score. The presence of aggressive behavior in schizophrenic patients indicates the severity of the disorder to some degree. NLR can be used as an objective biomarker to quickly assess the risk of aggression in schizophrenic patients.

## 1. Introduction

Schizophrenia is a complex illness with no recognized cause. The significant symptoms are affective disorders, association disorders, and volitional disorders [1]. Because schizophrenia's performance varies from patient to patient and at different times in the same patient, the disease's features are highly variable. Current treatment approaches and outcomes are inferior, putting a massive cost on society [2]. Thus, yet, there have been few studies on schizophrenia. Its diagnosis and evaluation are based mainly on a thorough medical history and mental status examination, with no specific laboratory markers or pathophysiological signs.

Aggressive behavior is a common characteristic of schizophrenia during acute episodes, and it poses a severe threat to the patient's and society's safety [3]. It is generally known that people with schizophrenia are more prone than the general population to engage in aggressive conduct at any time during their disease, which has significant implications for patient care and treatment and raises the risk of harm [4]. Exploring effective monitoring measures for violent behavior in schizophrenia patients is essential for clinical practice and improves patient prognosis.

Peripheral blood inflammatory indicators, such as C-reactive protein (CRP), interleukin 6 (IL-6), tumor necrosis factor (TNF), C-reactive protein-albumin ratio (CAR), neutrophil-albumin ratio (NAR), and NLR, are a popular topic of current research for a variety of disorders. Among these, NLR is a novel marker of inflammation derived from routine blood count tests. Its association with inflammation has been reported in inflammatory bowel disease [5], diabetes mellitus [6], irritable bowel disease (Gulali [7]), COVID-19 infection (G. [8]), thyroiditis (G. [9]), and other thyroid conditions [10].

Aggression has been proven to be substantially linked to levels of organismal inflammation in usually healthy human participants [11]. This link has been confirmed in a variety of psychiatric diseases. Plasma CRP and IL-6 levels were linked to violent behavior in psychiatric disorders, according to Coccaro et al. [12]. According to a recent study, the expression of the TNF pathway has also been linked to aggressive behavior in bipolar disorder [13]. In a separate study, researchers discovered a link between central nervous system CRP and aggression in people with personality disorders [14]. However, aggression in schizophrenia patients is caused by a complicated set of factors that have yet to be fully understood. The association between it and the level of inflammation are unknown.

CRP levels were found to be higher in persons with schizophrenia in previous studies, and they were connected to illness severity and recurrence ([15]; L. [16]). A recent study by Zhou et al. also found that NLR has been linked to the severity of schizophrenia (X. [17]). Other findings show that CAR and NAR are higher in patients with schizophrenia than in healthy subjects (Y. H. [18]). Considering the chronic inflammatory state appears to be connected to the onset of schizophrenia (L. [16] [19]), as a result, it is plausible to believe that violent conduct in schizophrenia patients is linked to the body's level of inflammation. Once this idea is proven, it will serve as a potential biological signal for early assessing impulsive risk in schizophrenic patients.

We studied the findings of the assessment of peripheral blood inflammatory cell levels and BPRS and MOAS to obtain insight into the association between aggressive behavior and the amount of inflammation and severity of clinical symptoms in schizophrenic patients. In schizophrenia patients, we discovered a link between neutrophil count, NLR, and aggressive behavior. And this relationship existed not just before treatment but also after four weeks of treatment. Because NLR is more stable than neutrophil count, it can be utilized as a potential biological marker to assess the risk of aggression in schizophrenia patients in a cost-effective, objective manner.

## 2. Methods

### 2.1. Study Overview and Participants

From September 2020 to April 2021, all subjects were admitted to The Affiliated Xuzhou Eastern Hospital of Xuzhou Medical University. The following criteria were used to determine eligibility: (1) meeting the diagnostic criteria for schizophrenia in the International Classification of Diseases, Tenth Edition (ICD-10); (2) age 18 to 65 years; (3) acute onset of illness; and (4) no antipsychotic or sedative-hypnotic drugs within six months of enrollment. The exclusion criteria are as follows: (1) severe brain disease, immune disease, or other physical severe diseases (heart disease, diabetes, thyroid disease, and other endocrine diseases); (2) infection, fever, or use of anti-inflammatory drugs, antibiotics, immune preparations, lithium carbonate, or other drugs that affect test results four weeks before enrollment; (3) lactating and pre-menopausal women; and (4) within a year, the participants reported using alcohol, narcotics, and other psychoactive substances.

### 2.2. Inspection Method

#### 2.2.1. Personal Characteristics Collection

The individuals' demographic information, such as gender, age, education, marriage, and occupation, were collected using a homemade general information questionnaire.

#### 2.2.2. Treatment Options

Given the minimal effect of aripiprazole on the degree of inflammation in the body of schizophrenia patients [20], all cases were treated with aripiprazole pills from Jiangsu Nhwa Pharmaceutical Co., Ltd. (production lot number AL200305). Begin with five milligrams per day and progressively increase to the lowest effective dose over two weeks. If necessary, benzodiazepines might be added to the treatment without using other antipsychotics.

#### 2.2.3. Evaluation of the Severity of Clinical Symptoms

The BPRS was used to assess the subjects' clinical symptoms [21]. The assessment items included 18 items: somatic concerns, anxiety, emotional withdrawal, conceptual disorganization, guilt feelings, tension, mannerisms and posturing, grandiosity, depressive mood, hostility, suspiciousness, hallucinatory behavior, motor retardation, uncooperativeness, unusual thought content, blunted affect, excitement, and disorientation. Each item is rated on a 7-point scale of not present, very mild, mild, moderate, moderately severe, severe, or extremely severe. It is widely used in China because it properly reflects the severity of psychiatric symptoms and has higher reliability and validity [22, 23]. Two trained physicians examined the study in a double-blind way, and the mean of the data was taken. We performed a test of agreement between the scores of the two evaluating physicians, with an intragroup correlation coefficient of ICC = 0.842.

#### 2.2.4. Aggression Assessment

The MOAS was used to evaluate subjects for aggressive behavior a week before their hospital admission. Yudofsky et al. [24] of Columbia University established the Overt Violence Scale (OAS) in 1984. It is extensively used to aid clinical recording and describe aggression in mental disease patients. However, algebraic accumulation was used to get the overall score for each form of aggressiveness on this scale, and the scores for diverse behavioral styles of aggression were the same. Kay et al. [25, 26] altered the OAS to address the scale's shortcomings. Verbal aggression, aggression against objects, aggression against oneself, and aggression against others are the four types of aggression identified by MOAS. Five ratings are given on a scale of 0 to 4, and specific behavioral patterns are defined. MOAS calculates weighted ratings for several sorts of aggressions as follows: verbal aggression × 1, aggression against objects × 2, aggression against self × 3, and aggression against others × 4. Because the final total score is the sum of all weighted values (max = 40), differing levels of aggression are more likely to be reflected in the final rating score. Professor Bin Xie of the Shanghai Mental Health Center translated the scale into Chinese in 1991, and it has intermediate reliability and validity in a sample of Chinese psychiatric inpatients [27]. It is extensively used in Chinese psychiatric medical and research institutions [28]. According to previous studies [29], the weighted total score is greater than or equal to 5 as the inclusion criteria for the “seriously aggressive” group was used to split the subjects into aggressive and nonaggressive groups.

#### 2.2.5. Blood Cell Analysis

At 6 : 30-7 : 00 am on day two and the 4th weekend after admission, 5 ml of elbow venous blood was collected under the fasting state of the subject and placed in an EDTA anticoagulation tube. Japan Sysmex Corporation provided the reagents, and the instrument was a Sysmex XN-1000 fully automated hematology analyzer developed by Japan Sysmex Corporation. Blood cell analysis was performed using a semiconductor laser and the resistive resistance method. The test results include WBC count, platelet count, neutrophil count, lymph count, monocyte count, eosinophil count, basophil count, and calculation of PLR, NLR, and MLR.

#### 2.2.6. Statistical Analysis

For statistical analysis, the SPSS 23.0 software package was employed. Kolmogorov–Smirnov test was used for normality analysis of the study variables. To compare general information, BPRS, and blood cell counts between the two groups, an independent sample *t* test was utilized. The BPRS, blood cell counts, and other outcomes were compared before and after therapy using a paired-sample *t* test. The relationship between aggressive behavior, BPRS, and blood cell counts was investigated using Spearman correlation analysis. A statistically significant difference was defined as *P* < 0.05.

## 3. Results

### 3.1. Subject Characteristics

The total number of subjects was 213. There were 72 cases in the aggressive group, including 28 males and 44 females aged 18-65, with a mean age of 41.57 ± 13.24 years. The nonaggressive group consisted of 141 cases, including 56 males and 85 females aged 18-65, with a mean age of 40.66 ± 12.63 years. There were no statistically significant differences between the two groups in age (*t* = −0.489, *P* = 0.625), gender (*χ*^2^ = 0.014, *P* = 0.907), education (*χ*^2^ = 5.299, *P* = 0.506), marital status (*χ*^2^ = 0.092, *P* = 0.993), and aripiprazole dose (*t* = 1.420, *P* = 0.157).

### 3.2. Comparison of BPRS Scores and Blood Cell Counts before and after Treatment between the Two Groups

Before treatment, there were statistically significant differences in total BPRS score, WBC count, neutrophil count, monocyte count, NLR, and MLR between the two groups. There were no statistically significant differences in platelet count, lymphocyte count, eosinophil count, basophil count, and PLR (Table 1).

One case in the nonaggressive group was shed due to refusal to review blood cell analysis at the end of the fourth week of treatment and inability to complete the study. In Table 2, the differences in the total BPRS score and neutrophil count between the two groups after treatment were statistically significant. The differences between WBC count, platelet count, lymphocyte count, monocyte count, eosinophil count, basophils, PLR, NLR, and MLR were not statistically significant.

### 3.3. Correlation Analysis of Aggressive Behavior with BPRS and Blood Cell Count before and after Treatment

Correlation analysis showed that subjects' pretreatment aggressive behavior was positively correlated with BPRS total score, WBC count, neutrophil count, monocyte count, NLR, and MLR. There was no significant correlation with platelet count, lymphocyte count, eosinophil count, basophil count, and PLR.

Aggressive behavior was positively correlated with total BPRS score, neutrophil count, and NLR at the end of 4 weeks of treatment. There was no significant correlation with WBC count, platelet count, lymphocyte count, monocyte count, eosinophil count, basophil count, PLR, and MLR (Table 3).

## 4. Discussion

Earlier studies have shown that the incidence of aggressive behavior in patients with schizophrenia is significantly higher than in the general population [30]. This study investigated the aggressive behavior of 213 patients admitted in the acute phase of schizophrenia and found the prevalence of aggressive behavior to be 33.94%. This result is consistent with Wen Li et al. [31] and warrants great concern. People with schizophrenia tend to use psychoactive substances frequently, have psychopathy, and have thoughts of persecution, so they are prone to aggressive behavior [32]. As a result, health-care personnel should take steps to minimize their hostile and violent behavior toward others.

In recent years, the hypothesis of inflammatory mechanisms in schizophrenia has received increasing attention from researchers. Both animal and clinical studies suggest that the onset of schizophrenia is closely related to the level of inflammation in the body [33–35]. People with high levels of immunological and inflammatory markers are at a higher risk of developing schizophrenia. Furthermore, people with high levels of inflammatory substances are more prone to create neurocognitive impairment, leading to psychotic symptoms. There is an interaction between psychiatric symptoms and inflammatory substances [36]. Another study found that patients with schizophrenia and at-risk groups have problems with their innate and adaptive immune systems. Immune dysfunction may play a role in the pathogenesis of schizophrenia, and its clinical symptoms may be potentially associated with the levels of inflammatory cytokines that regulate the immune response (G. M. [37]; Golam M [38]). In this study, the level of inflammatory cells in the blood reduced as the BPRS score decreased following therapy in both the aggressive and nonaggressive groups. This result supports the findings of Xia Zhou et al. [17], indicating that the amount of organismal inflammation may reflect the condition of patients with schizophrenia in the acute phase to some extent.

However, the association between schizophrenic patients' aggression and their body's level of inflammation is still unknown. In some studies, C-reactive protein levels were associated with schizophrenia aggression ([39] [16]). Sourav et al. [40] showed that interferon-gamma (IFN-G) and interleukin 10 (IL10) were strongly associated with aggressive behavior in schizophrenia. According to a recent study, CAR may predict a distinct tendency to fatal aggression in schizophrenia as a proxy marker of peripheral inflammation (Yasin Hasan [41]). However, the biomarkers mentioned in the above study are not routine clinical tests and cannot be tested in most basic hospitals. To find a simple, stable, and easily detectable biomarker to assess the risk of aggression in schizophrenia, we performed an in-depth analysis of the results of blood cell analysis in subjects. NLR is an essential indicator of inflammation in the body. It is widely used in atherosclerosis [42], cardiovascular disease, and other [43] inflammatory diseases. Previous studies have found an association between NLR and the severity of schizophrenia [44], but no relationship has been reported between it and the risk of schizophrenic aggression. Our study found that neutrophil count and NLR were not only positively correlated with aggressive behavior in schizophrenic patients before treatment, but this correlation persisted after treatment. Considering that NLR is a ratio of neutrophils to lymphocytes, it is more stable than a single neutrophil count. Therefore, NLR can be used as a potential biomarker to assess aggressive behavior in schizophrenic patients.

Aggressive conduct can develop for a variety of causes in people with schizophrenia. Coccaro et al. [14] found that inflammatory proteins in the cerebrospinal fluid increase phagocytosis, activate complement, and induce the release of proinflammatory cytokines. Inflammatory processes that persist cause cellular damage in the brain and elsewhere. These inflammatory activities play a crucial role in regulating aggressive behavior. A similar discovery was made by Barzilay et al. [39]. According to Fanning et al. [45], childhood abuse has a considerable impact on violent and aggressive conduct in adult schizophrenics. Because childhood stress can impact the inflammatory response, aggressive behavior is regulated indirectly. The causes of aggressive conduct in schizophrenia patients are, of course, complicated. They include the following risk factors: substance abuse, physical or sexual abuse, hallucination/delusional beliefs, poor insight, poor impulse control [46], gender, age, literacy [47], hormone levels, neurotransmitters (dopamine and 5-HT), lipoprotein abnormalities [48], neurogenic trophic factor, and cytokine interactions [49, 50]. Therefore, it is not possible to attribute all aggressive behavior in schizophrenia to the high inflammatory level of the organism on only one hand.

In conclusion, in this study, we found that patients with schizophrenia had a high incidence of aggressive behavior. The level of inflammation in the organism of schizophrenic patients decreases as the disease goes into remission. Further investigation revealed that NLR was positively connected with aggressive behavior in schizophrenic patients both before and after treatment, suggesting that it could be used as a biological indicator to predict aggressive behavior in schizophrenic patients. Our study has added to our knowledge of the potential link between schizophrenic aggression and inflammation. The test for inflammatory cells in the peripheral blood is affordable, easy to do, and has long been widely performed in many primary care institutions. The findings of this study make it easier for medical practitioners to employ simple laboratory instruments to analyze the level of inflammation (acquisition of NLR) in patients with schizophrenia and initial screen for and assess the risk of schizophrenia aggression using NLR as a biomarker.

Limitations of this study are as follows: (i) the relatively small sample size of this study may reduce statistical efficacy; (ii) all subjects were treated for only four weeks, and the long-term relationship between inflammation levels and aggression could not be assessed; and (iii) plasma inflammatory cytokine levels are not specific indicators and are influenced by a variety of factors, such as body mass index (BMI) [51], antipsychotics [52], and smoking [53]. In this investigation, these factors were not strictly controlled, which could have influenced the outcomes.

## Figures and Tables

**Table 1:** Comparison of BPRS and blood cells before treatment in the two groups ($\overset{-}{x}\pm s$).

	Aggressive behavior group (*n* = 72)	Nonaggressive behavior group (*n* = 141)	*t*	*P*
BPRS	71.64 ± 11.23	52.62 ± 4.61	-13.792	≤0.001
WBC	7.38 ± 1.79	6.71 ± 1.85	-2.536	0.012
Platelet	244.46 ± 67.13	229.75 ± 56.28	-1.688	0.093
Neutrophils	4.66 ± 1.65	4.04 ± 1.62	-2.596	0.010
Lymph	2.02 ± 0.74	2.02 ± 0.62	-0.065	0.949
Monocyte	0.57 ± 0.17	0.51 ± 0.16	-2.619	0.009
Eosinophils	0.12 ± 0.10	0.11 ± 0.10	-0.274	0.784
Basophils	0.02 ± 0.01	0.02 ± 0.01	-0.141	0.888
PLR	139.59 ± 79.01	124.95 ± 55.23	-1.407	0.162
NLR	2.73 ± 1.78	2.20 ± 1.23	-2.268	0.025
MLR	0.32 ± 0.14	0.27 ± 0.10	-2.507	0.014

**Table 2:** Comparison of BPRS and blood cells after treatment in the two groups ($\overset{-}{x}\pm s$).

	Aggressive behavior group (*n* = 72)	Nonaggressive behavior group (*n* = 140)	*t*	*P*
BPRS	33.32 ± 6.32	29.51 ± 6.19	-4.215	≤0.001
WBC	6.71 ± 1.74	6.29 ± 1.62	-1.755	0.081
Platelet	241.39 ± 59.39	228.69 ± 55.84	-1.535	0.126
Neutrophils	4.00 ± 1.50	3.57 ± 1.30	-2.151	0.033
Lymph	2.02 ± 0.61	2.04 ± 0.59	0.204	0.839
Monocyte	0.52 ± 0.15	0.49 ± 0.16	-1.379	0.169
Eosinophils	0.14 ± 0.10	0.16 ± 0.12	0.766	0.444
Basophils	0.03 ± 0.05	0.03 ± 0.02	-1.482	0.140
PLR	130.31 ± 52.54	121.57 ± 45.28	-1.259	0.209
NLR	2.16 ± 1.04	1.92 ± 1.07	-1.546	0.124
MLR	0.28 ± 0.13	0.25 ± 0.10	-1.673	0.097

**Table 3:** Correlation analysis between aggression and BPRS and blood cells before and after treatment (*r*).

	Aggression	
	Before treatment (*n* = 213)	After treatment (*n* = 212)
BPRS	0.806^**^	0.237^**^
WBC	0.177^**^	0.115
Platelet	0.094	0.086
Neutrophils	0.191^**^	0.140^*^
Lymph	-0.016	-0.038
Monocyte	0.165^*^	0.113
Eosinophils	0.023	-0.031
Basophils	0.033	0.118
PLR	0.063	0.077
NLR	0.146^*^	0.137^*^
MLR	0.146^*^	0.095

^*^ *P* < 0.05. ^**^P < 0.01.

## Data Availability

The data used to support the findings of this study are available from the corresponding author upon request.
